The article "Phase Prediction Study of High-Entropy Energy Alloy Generation Based on Machine Learning" was retracted in 2022. Reason: concerns about the peer review.

# Phase Prediction Study of High-Entropy Energy Alloy Generation Based on Machine Learning

**DOI:** 10.1155/2022/8904341

**Published:** 2022-06-06

**Authors:** Zhongping He, Huan Zhang

**Affiliations:** School of Mechanical Engineering, Chengdu University, Chengdu 610106, Sichuan, China

## Abstract

Traditional energy sources such as fossil fuels can cause environmental pollution on the one hand, and on the other hand, there will be a shortage of diminishing stocks. Recently, a variety of new energy sources have been proposed by scientists, such as nuclear energy, hydrogen energy, wind energy, water energy, and solar energy. There are already many technologies for converting and storing energy generated from new energy systems, such as various storage batteries. One of the keys to the commercialization of these new energy sources is to explore new materials. Researchers have performed a lot of research on new energy material preparation, mechanical properties, radiation resistance, energy storage, etc. However, new energy metal materials are still unable to combine radiation resistance, good mechanical properties, excellent energy storage, and other characteristics. There is still a lack of breakthrough materials with better performance or more stable structure. Recently, researchers have discovered that high-entropy alloys have become one of the most promising new energy metal materials. Because it not only has high energy storage and high strength, but also has high stability and high radiation resistance, and is easy to form a simple phase, the prediction of phases in high-entropy energy alloys is very critical, and the generation of designed phases in high-entropy energy alloys is a very important step. In this study, three machine learning algorithms were used to predict the generated phase classification in high-entropy alloys, namely, support-vector machine (SVM) model, decision tree (DT) model, and random forest (RF) model. The models are optimized by grid search methods and cross-validated, and performance was evaluated with the aim of significantly improving the accuracy of generative phase prediction, and the results show that the random forest algorithm has the best prediction ability, reaching 0.93 prediction accuracy. The ROC (receiver operating characteristic) curve of the model shows that the random forest algorithm has the best classification of solid-solution (SS) phases, where the classification probabilities AUC (area under the curve) area for amorphous phase (AM), intermetallic phase (IM), and solid-solution phase (SS), respectively, are 0.95, 0.96, and 1, respectively, , which can predict the generated phases of high-entropy energy alloys well.

## 1. Introduction

With economic development, world energy consumption is exponentially growing and is expected to reach 28TW by 2050, which is a total of 20 billion tons of oil consumed every year [1]. The combustion of fossil fuels produces greenhouse gases, and the emission of these greenhouse gases can lead to serious environmental problems, not only in terms of air pollution, such as emissions from car exhaust, but also in terms of global warming [2]. Fossil fuels are also limited on Earth and cannot be used forever. All of these act as a limit to the use of fossil fuels. Currently, fossil fuels account for about 95% of global energy consumption [3], and eliminating this problem will require a transition to reliable, renewable, and green energy sources, such as hydropower, solar energy, and wind. This transformation is possible even today, but most renewable energy sources are not continuously powered, such as solar panels when there is no sun and wind turbines when there is no wind. Therefore, energy storage mechanisms and energy conversions need to be more and more efficient than before, which require continuous research and development. In addition, capturing and converting carbon dioxide are a possible option for reducing greenhouse gas emissions and producing carbon-based fuels. The research of advanced high-entropy alloy materials is conducive to the realization of these beautiful ideas. In recent years, hydrogen storage high-entropy alloys, battery high-entropy alloys, and nuclear power high-entropy alloys are receiving increasing attention [4, 5]. Lattice distortion is prevalent in high-entropy alloys, and because better reactive sites are formed, the lattice distortion facilitates gas absorption, resulting in good hydrogen storage properties. The binder-free electrode is made of high-entropy alloy, which not only has a high-capacity capacitance of 700 F cm^−3^ but also has an excellent cycle stability of more than 3,000 cycles. These excellent properties are far superior to the latest research on nanoporous metals. High-entropy alloys can be used as both radiation-resistant materials in the nuclear industry and high-temperature materials in aerospace engineering, with multiple potential applications in extreme environments.

Current methods of the preparation of high-entropy energy alloys include the melt-casting method, powder metallurgy method, melt-spinning method, and deposition technique method. The manufacturing cost, processing capability, and complexity of experiments in the preparation of high-entropy energy alloys often make the fabrication of high-entropy energy alloys hindered, and it is difficult to obtain the desired results. Due to the complex elemental composition of high-entropy energy alloys, the calculation of high-entropy energy alloys using conventional methods is not only difficult and expensive, but the diversity of influencing factors also adds difficulties to the design of high-entropy energy alloys, whose excellent properties depend on the composition of the generated phases, so the accurate prediction of the generated phases of high-entropy energy alloys is crucial to the development and application of high-entropy energy alloys.

As a part of artificial intelligence, machine learning combines machine learning techniques with material science to take full advantage of data-driven technologies, and gives new means and directions to materials science research. Data can be obtained from various material databases, experiments, and material simulation calculations, and data mining can be performed using machine learning. More and more researchers are now turning their attention to this new way of research, and the number of machine learning-assisted material design in materials science is growing at an alarming rate.

Zhang et al. [6] studied the thermodynamic properties of high-entropy alloys through Monte Carlo simulations. By taking the pairwise interactions between atoms as characteristic parameters, the representativeness of the dataset is systematically improved. In the process of designing high-entropy alloys with Monte Carlo simulation, a reliable theoretical basis can be obtained through sample application. But since this process is not only very complex, but also time-consuming and inefficient, the above case only works for simple cases. Thermo-Calc uses the CALPHAD method to assist in predicting performance metrics, but determining this field requires significant experimental and computational costs. A method to obtain high-strength and low-cost medium-entropy alloys based on the combination of high-throughput experiments and simulation calculations with machine learning was proposed by Li et al. [7], which provided ideas and references for later scholars. Improving the design of high-entropy alloys by exploiting the electronic parameters of the alloy (electronegativity, valence electron concentration, etc.) was proposed by Poletti et al. [8]. But this method predicts less accuracy. An approach that combines the application of machine learning (ML) from thermodynamic data and composition-based features was proposed by Kaufmann and Vecchio [9], which enables fast searches for single-phase solid solutions. Miracle [3] found that the large composition space offers opportunities to improve properties such as hardness, but there are still problems in composition optimization that are still problematic, especially if explored by “trial and error” or intuition.

Islam et al. [10] used an artificial neural network to make predictions in multiprincipal element alloy phases. He used about 118 components as a dataset and found that the artificial neural network had an average prediction accuracy of 80%. Huang et al. [11] performed phase classification on a dataset with five input features for three-stage (AM, IM, and SS) classification, and the best K-nearest neighbor (KNN), support-vector machine (SVM), and artificial neural network(ANN) results were 68.6%, 64.3%, and 74.3%, respectively, indicating that artificial neural network is the best classification algorithm. Zhou et al. [12] applied three different machine learning algorithms (ANN, SVM, and KNN) for the phase prediction of high-entropy alloys. The feature set in this study contains 13 parameters, respectively, melting temperature mean and standard deviation of atomic size, mean and standard deviation of atomic size, mean and standard deviation of mixing enthalpy, mean and standard deviation of ideal mixing entropy, mean and standard deviation of electronegativity, and mean and standard deviation of valence electron concentration (VEC). The models with reduced features were verified to perform worse than those with complete features by means of feature reduction techniques. Zhang et al. [13] selected machine learning models and descriptors by using a genetic algorithm, and applied the algorithm to two classification problems, one is face-centered cubic (FCC), body-centered cubic (BCC), and biphasic, and the other is the solid solution (SS) and nonsolid solution (NSS). For the first classification problem, the support-vector machine using the radial basis function (RBF) algorithm has the best classification performance, with a test accuracy of 88.7%. For the second classification problem, the neural network algorithm was 91.3% accurate. Two machine learning algorithms (DT and RF) for high-entropy alloy phase classification (FCC + BCC SS, BCC SS, FCC SS, and IM) were evaluated by Machaka [14]. The input feature set consists of five eigenvalues. The research results show that random forest achieves good results in phase classification, with a test accuracy rate of 82.3%. Roy et al. [15] used ML models to forecast the crystalline phases and Young's modulus for high-entropy alloys, medium-entropy alloys, and low-entropy alloys composed of five refractory elements, and finally obtained that electronegativity difference and the average melting point of the elements are important influencing factors for the formation of alloy phases, and melting temperature and mixing enthalpy are influencing Young's modulus for these materials. The key factors affecting Young's modulus of these materials are the melting temperature and the mixing enthalpy. The work related to the prediction of the generated phases of high-entropy alloys by ML techniques has been successively reported, but for the more important phase properties of high-entropy alloys, there are still problems such as few empirical parameters adopted for the generated phases of alloys, the low prediction accuracy of machine learning models, poor generalization ability, and low learning efficiency. Mamun et al. [16] built a variational autoencoder-based generative model by conditioning on the experimental dataset to sample hypothetical synthetic candidate alloys. A gradient boosting algorithm is used to train ML models for very accurate prediction of rupture life in a variety of alloys.

Machine learning-based research on high-entropy alloys [6–16] has largely helped the materials' discipline to reduce a lot of unnecessary time and costs. However, many algorithms do not achieve the expected results, and the prediction results can only reflect the results of a certain aspect, for the lack of data and data incompleteness. The use of multiple features in combination leads to prediction results and expectations that are very different. In the current materials' discipline, there is no complete system for high-entropy alloys, and the factors affecting them cannot be fully considered. There are often more extreme scenarios based on a single influencing factor to predict multiple influencing factors together, and they fail to consider that the factors affecting different phases are also different. Different algorithms are used to address this issue of a single phase to be relevant, rather than a single description of an algorithm to solve the problem that has better value.

In this study, three different ML models, such as support-vector machine (SVM), decision tree (DT), and random forest (RF), are used to forecast the phase to produce of high-entropy energy alloys, as shown in Figure 1, and the different models are optimized using cross-validation and grid search, and finally, the model is evaluated using ROC curves, which leads to the prediction of the generated phases of high-entropy alloys for biomedical applications.

## 2. Machine Learning Algorithms

### 2.1. Support-Vector Machine (SVM) Algorithm

Support-vector machines (SVMs) are one of the most popular models in the domain of ML model and are loved by a large number of machine learning researchers. This entirely depends on its powerful capabilities to handle almost any problem that is not well handled or cannot be handled by other models. The model is very suitable for datasets that are not too complex and are around small to medium in size to achieve more desirable results. Support-vector machines specifically often handle the following tasks: linear or nonlinear classification, regression, and outlier detection classification. Linear classification uses a straight line to separate different categories (same categories are grouped together), and the separated categories will move away from this line, which is called the decision boundary. Linear regression in particular requires feature scaling, without which the prediction results are often very poor. Because many datasets are not linearly separable, there is no way to use linear means of classification but rather nonlinear. The main solution for nonlinear classification is to add polynomial features to the dataset (e.g., transforming a 1D dataset into a 2D dataset) so that the nonseparable becomes a separable problem, which can then be solved. There is another solution, which is to add similar features and use the Gaussian radial basis function as the similarity function. By performing calculations with this function, new similar features can be obtained, and after transforming the dataset, they also become separable.

### 2.2. Decision Tree (DT) Algorithm

A decision tree (DT) is also a kind of ML model algorithm, which is also an important part of a random forest algorithm, and its purpose is to get a decision tree with strong generalization ability, that is, excellent prediction ability for uncertain material. The basic idea of the decision tree is executed based on the idea of a tree structure. Taking binary classification as an example, a model is trained from a given dataset and used to classify new data. How to choose the optimal division attributes is significant trouble to be resolved by the decision tree algorithm. That is, the branch structure of the decision tree contains as many nodes of the same class as possible, i.e., the “purity” of the nodes is high. There are several ways to select the best way to classify attributes, such as information entropy and information gain. The overall structure of the decision tree algorithm is divided into three parts, namely, the root node, the internal node, and the leaf node, of which there is only one root node, and other nodes can contain infinite nodes. The root node performs the input of processed data samples, the internal nodes perform the attribute testing also called attribute filtering, and the leaf nodes correspond to the decision results. The implementation process is to input the entire dataset to the root node, and then, the decision tree algorithm uses the optimal attribute division to do further division for each branch node (if more than one optimal attribute is obtained, then one of them is selected) from the root node to each leaf node that belongs to a decision path.

### 2.3. Random Forest (RF) Algorithm

Random forest (RF) algorithm = bagging (resampling) + decision tree. The basic principle is as follows: the combination of multiple classifications and regression tree (CART) (CART trees for the use of GINI algorithm decision tree). To significantly improve the final result, randomly assigned training data need to be added, by combining many “feeble learners” in order to build a powerful model: a “strong learner.” This approach is also known as the integration approach, which is the concept of “three stinkers are better than one.” However, there is only one dataset, so to form multiple trees with differences for the integration method, it is necessary to generate different datasets in order to produce multiple CART trees with differences, and there are two ways to do it: (1) bagging (bootstrap aggregation). Bootstrap means “resampling the original data to produce new data, the sampling process is uniform and repeatable”; using bootstrap can generate multiple datasets from a set of data. This method extracts K samples from the training dataset and then trains K classifiers from these K samples. The K samples are put back into the parent each time, so some of the information will be duplicated among the K samples, but since each tree has different samples, the trained classifiers (trees) are different from each other, and the weights of each classifier are the same. (2) boosting. Similar to bagging, but with more emphasis on studying the error part to boost the gross efficiency. The training of the new classifier is achieved by increasing the proportion of erroneous data related to the previous classifier and increasing the training of the wrong part. Through such an exercise, the new classifier will learn the features of the wrong data and will not export the wrong features, thereby improving the results of the classifier's prediction.

## 3. Simulation of Phase Structure of High-Entropy Energy Alloys

### 3.1. Data Collection

Through the existing literature [3, 9–15], the phase structure law of high-entropy energy alloys is understood. The relevant parameters involved in the formation of high-entropy energy alloy phases were also investigated. Relevant data parameters were collected, and a total of 325 high-entropy alloy data were obtained. By removing redundant data and initially cleaning the data, a dataset containing 293 alloy data was finally formed, which included 72 solid solutions (SSs), intermetallic compounds (IM) 163, and amorphous (AM) 92. The valence electron concentration (VEC), mixing enthalpy (Δ*H*_mix_), mixing entropy (Δ*S*_mix_), atomic radius difference (*δ*), the average melting point of constituent elements (*T*_melt_), and electronegativity difference (Δ_*χ*_) are selected as the input of machine learning, and the feature variables and their formulas are shown in the following equations, with the classification of the generated phases of high-entropy energy alloys as the output of machine learning, which is the target variable.

(1) $$\begin{array}{c} \delta =\sqrt{\sum_{i=1}^{n}ci{\left(1-\frac{ri}{a}\right)}^{2}},\\ T_{\text{melt}}=\sum_{i==1}^{n}c_{i}T_{mi},\\ \Delta H_{\text{mix}}=4\sum_{i\neq j}c_{i}c_{j}H_{ij},\\ S_{id}=-k_{B}\sum_{i=1}^{n}c_{i}\ln\;c_{i},\\ \chi =\sum_{i=1}^{n}c_{i}\chi_{i},\\ \text{VEC}=\sum_{i=1}^{n}c_{i}{\text{VEC}}_{i}. \end{array}$$

In the above equation, *δ* is atomic radius difference; *C*_*i*_ is atomic concentration of *i* element; n is amount of elements in metal; *r*_*i*_ is atomic radius of the *i* element; a is average atomic radius; *T*_*mi*_ is melting temperature of the *i* element; *T*_melt_ is average melting temperature of the metal; *H*_*ij*_ is enthalpy of atomic pairs calculated with Miedema's model; Δ*H*_mix_ is enthalpy of blending of elements *i* and *j*; *k*_*B*_ is Boltzmann constant; *S*_*id*_ is the ideal mixing entropy; *χ*_*i*_ is electronegativity of element *i*; and VEC_*i*_ is valence electron concentration of element *i*.

### 3.2. Software Selection

This experiment is based on Python 3.8 for data processing and model building, using Python as the programming language and Jupyter Notebook as the development tool, with its powerful visualization interface, which brings great convenience for data processing. The open-source library sklearn 0.24 was used to complete the classification task. Sklearn library is, respectively, divided into six major parts: regression task, clustering task, dimensionality reduction task, model selection, and data preprocessing. This study mainly uses the classification model random forest (RF) and decision tree (DT) to complete the high-entropy alloy phase classification problem.  Table 1 is to apply the pandas model in Python to display part of the information.

### 3.3. Data Processing

When training with support-vector machines (SVMs) for high-entropy alloy data, the data need to be normalized. In this study, in order to control the eigenvalue of each feature between 0 and 1, the pandas library achieves the purpose through the following relationship, calculated as shown in the following equation.

(2) $$\begin{array}{c} X_{\text{new}}=\frac{X_{i}-X_{\min,i}}{X_{\max,i}-X_{\min,i}}, \end{array}$$

where *X*_new_ is the normalized feature, and *X*_*i*_ is primary data from one of the five characteristics. *X*_max,*i*_ and *X*_min,*i*_ are the maximum and minimum values of features, respectively. Dimensionless numerical features are generated through a normalization process. This process ensures that each numerical feature has the same numerical scale and that all numerical features are fairly treated, which is also more conducive to the training model, making it ultimately more accurate in terms of prediction accuracy.

### 3.4. Model Evaluation

In the training process, the training and test sets used are for the classification problem. For classification problems, machine learning usually uses precision, recall, F1 value, accuracy, error rate, and ROC (receiver operating characteristic) curves as classification metrics. In this current research, the K-fold cross-validation method was used to continuously optimize the model, prevent data overfitting, divide the training data and test data, and verify the accuracy of the model. The 10-fold cross-validation method is used, in which the experimental data are divided into 10 groups, of which 9 groups are used for training the model and 1 group is used for validation, and the accuracy of the algorithm is estimated by averaging the 10 eigenvalues. In the later validation of the model performance, the prediction performance of the algorithm model was evaluated by plotting ROC-AUC curves; first, all samples were sorted by prediction probability, and the corresponding FPR and TPR were calculated using the prediction probability of each sample as the threshold and then connected by line segments. The calculation process is shown in the following equation, where *X* are Y are denoted as horizontal coordinates and vertical coordinates, respectively. FPR is the probability of incorrect samples being classified as correct, and TPR is the probability of correct samples being classified as correct.

(3) $$\begin{array}{c} X:\text{FPR}=\frac{\text{FP}}{\text{FP}+\text{TN}},\\ Y:\text{TPR}=\frac{\text{TP}}{\text{TP}+\text{FN}}, \end{array}$$

where FP (false positive) means that the actual fraudulent specimen is forecasted as honest specimen; TN (true negative) means that the actual honest specimen is forecasted as honest specimen; TP (true positive) means that the actual fraudulent specimen is forecasted as fraudulent specimen; and FN (false negative) means that the actual honest specimen is forecasted to be a fraudulent specimen. As the area under the ROC curve, AUC, it is between 0.1 and 1. The value of AUC can intuitively evaluate the quality of the classifier. The closer the value of AUC is to 1, the better the classification effect of the classifier.

## 4. Discussion

In this study, feature importance is optimized by using the open-source machine learning library scikit-learn, using the random forest classifier algorithm. Then, their importance is ranked and it is found that the importance of both mixed entropy (ΔS, Sid) and atomic radius difference (*δ*, delta) is relatively low, as shown in Figure 2, the important coefficient of mixed enthalpy (ΔH) reaches 0.35, and the coefficient of atomic radius difference is 0.08.

To visualize feature importance and to understand the correlation between two and two features, a scatter plot of the three stages between two and two feature factors was plotted in this study, as shown in Figure 3. In this plot, the correlation between two features, *H*_mix_ and D_Tm, is clearly shown, and to some extent, there is a boundary to separate them. However, for the correlation analysis of VEC and delta, the boundary that separates these phases becomes blurred. Based on this figure, it can be inferred that *H*_mix_ and D_Tm are the most important features in this study. Meanwhile, the diagonal subplot shows the histogram of the phase distribution. As can be seen from Figure 3, all histograms in any of the subplots in Figure 3 cannot be separated from each other, which means that there is no single feature that can be used to fully classify the high-entropy alloy phases.

In this study, three machine learning algorithms introduced above, including RF classifier, SVM classifier, and DT classifier in the scikit-learn library, are used to establish the model. To fully use the training set or validation set, the training process uses the 10-fold cross-validation method to train the data, and the training accuracy is shown in Table 2. To prevent data overfitting, the collected experimental data are divided into two groups, one is training data and the other is test data, of which 9 groups of experimental data are used as training data and 1 group of experimental data is used as test data. Each algorithm was trained 10 times according to the same method, and algorithm accuracy is assessed by averaging ten feature values. The average evaluation accuracy of the three algorithms is displayed in Figure 4 below, in which the SVM (support-vector machine) classifier and the random forest classifier, respectively, achieved a prediction accuracy of 0.88 and 0.82.

In the classification decision tree used in this study, using information gain as a criterion for finding leaf nodes, the maximum depth used in this study is 9. If the depth is very large, it leads to overfitting, while if the value of the depth value is too low, it leads to underfitting. During the training process in this study, the model training characteristic parameters were adjusted by the grid search method, showing the greatest deepness value of 9. The average cross-validation score with 10 groups for cross-validation was 0.78, and the prediction accuracy was achieved after constant tuning of the parameters, which means that the prediction of the classification formed by the phase using the decision tree classifier can be achieved for the data of the already existing high-entropy alloy. Similarly, in the random forest classifier study, parameter variations of *n* classification evaluators were used, and the values of the *n* estimators varied between 10 and 200 with an interval of 50, and the maximum deepness varied between 3 and 14. In this study, the greatest parameter value for the *n* estimators was 50 and the maximum depth was 13. The prediction accuracy for the best parameter value reached 0.91. In the support- vector machine algorithm, the radial kernel function was used as the kernel function for the classifier and the data were invariantly steeled to obtain a final prediction accuracy of 0.92.

To further assess the model performance and contrast the advantages and disadvantages of the three machine learning models, the ROC curve was also plotted in this study, and the prediction performance of machine learning algorithms for different generated phases of high-entropy alloys was evaluated by calculating the AUC area, as shown in Figure 5. Different machine learning models have different prediction ability for the generated phases of high-entropy alloys, DT is more inclined to the prediction of IM, RF is more sensitive to the formation of SS of high-entropy alloys, SVM is more favorable to predict AM, and for the overall prediction effect, the random forest has the best prediction ability, reaching a prediction accuracy of 0.93.

The refractory high-entropy alloy Ti-Zr-Nb-Mo system alloy was selected as the test set, and the best-performing random forest (RF) classifier was used to predict its generated phase. It was predicted to be a solid-solution (SS) phase for the Ti-Zr-Nb-Mo system refractory high-entropy alloy, which is the same as the experimentally measured data in other study. It fully demonstrates the reliability of the random forecast model to predict the generated phase of the high-entropy energy alloy.

## 5. Conclusions

In this study, three machine learning models were used to predict different generated phases of high-entropy alloys. The results of the analysis are summarized that different machine learning algorithms have different prediction results for the generated phases of high-entropy alloys, among which the RF model has the greatest manifestation with a precision of 0.93, while the ROC curve of RF training data is relatively smoother. In addition, because the parameters used in the model training process as the input to machine learning are random, the prediction results for different phases of the high-entropy alloy in the same machine learning model are different, among which RF has the best prediction for SS. In this study, machine learning is applied to the domain of high-entropy alloys to solve their phase classification problem and provide a possibility to find ideal high-entropy energy alloy components.

## Figures and Tables

**Figure 1:** Machine learning-based material development framework.

**Figure 2:** Feature ranking by random forest algorithm.

**Figure 3:** Scatter plot of the three stages between two feature factors.

**Figure 4:** Average evaluation accuracy of different algorithms.

**Figure 5:** ROC curves of three machine learning models.

**Table 1:** The six eigenvalue data used in this work in pandas module.

ALLOY	DELTA	D_TM	HMIX	SID	D_ELEC_NEGA	VEC	PHASE
B6NI21TA2	0.158000	438.290000	−23.258000	0.744100	0.122800	8.206900	IM
AL2B6CO20	0.161600	343.000000	−18.571400	0.758900	0.102300	7.285700	IM
B4INNI15	0.162200	397.070000	−13.380000	0.687400	0.062000	8.250000	IM
ALB2NI7	0.159300	371.510000	−19.600000	0.801800	0.111200	7.900000	IM
B6NI20TI3	0.165268	248.256278	−28.651605	0.816915	0.132398	7.931034	IM
…	**…**	**…**	**…**	**…**	**…**	**…**	**…**
ALER2	0.092700	394.340000	−33.777800	0.636500	0.174400	3.000000	IM
CE65AL12.5NI12.5CU10	0.148668	236.180373	−28.135000	1.030128	0.334994	4.675000	AM
CE65AL10NI10CU10NB5	0.144722	408.836767	−19.860000	1.120571	0.325392	4.600000	AM

**Table 2:** The 10-fold cross-validation method.

Model	10-fold cross-validation method									
SVM	0.700	0.900	0.800	0.966	0.966	0.931	0.828	1.000	0.828	0.966
DT	0.533	0.900	0.733	0.793	0.931	0.931	0.724	0.793	0.828	0.690
RF	0.567	0.900	0.767	0.931	0.862	0.896	0.689	0.827	0.758	0.931

## Data Availability

No data were used to support this study.
